This article has been retracted.

# Visual Dissemination of Intangible Cultural Heritage Information Based on 3D Scanning and Virtual Reality Technology

**DOI:** 10.1155/2022/8762504

**Published:** 2022-09-25

**Authors:** Wulong Xu, Xijie Sun, Shihui Pan

**Affiliations:** School of Journalism and Communication, Huanggang Normal University, Huanggang, Hubei 438000, China

## Abstract

In order to meet the needs of modern people for the acquisition of intangible cultural heritage information, the authors propose a research method that combines 3D scanning and virtual reality technology. Taking the production process of Xiuyu as an example, using Unity3D virtual reality technology combined with a digital platform, 3D modeling of Xiuyu is carried out, so that people can view the intangible cultural heritage information intuitively. The experimental results show that after using this method, more than 60% of more than 1000 people surveyed in the questionnaire want to experience intangible cultural heritage. In a survey of visualization platforms conducted at the same time, 90% of users are willing to combine jade carving technology with 3D scanning virtual reality technology. *Conclusion*. 3D scanning and virtual reality technology can further promote the process of inheritance and dissemination of intangible cultural heritage, accelerate the cultivation of intangible cultural heritage talents through the visualization platform, and promote the sustainable development of intangible cultural heritage, in order to better pass down the life memory and cultural genes of our ancient nation.

## 1. Introduction

With the changes in production and lifestyle in modern society, the living soil of intangible cultural heritage has undergone major changes and is now facing a rapid decline. The data shows that there are currently 1082 representative inheritors of intangible cultural heritage in my country, with an average age of 63 years, and only 7 young adults under the age of 40 inheritors, as shown in Figure 1. It can be seen that the national intangible cultural heritage has been aging; if the inheritance of intangible cultural heritage is weak, then some handicrafts inherited by word of mouth and behavior will gradually be forgotten by people; the traditional skills mastered by the old artists will not be inherited and practiced, and the national intangible cultural heritage culture will eventually disintegrate or even die out.

Therefore, innovative exploration of the inheritance and dissemination of intangible cultural heritage can make intangible cultural heritage play a more important role in national development, international social exchanges, and sustainable social development; this will further enhance the cultural self-confidence of the nation. Using the visualization platform as the communication medium, explore the feasibility and necessity of the application of digital technology in the inheritance and dissemination of intangible cultural heritage. Using virtual reality technology for “real” reproduction of intangible cultural heritage jade craftsmanship allows users to immensely experience traditional technological processes and processing methods and explore other new modes of inheritance and dissemination of intangible cultural heritage from point to point.

Changes in the media environment and the popularity of new communication methods have led to changes in information transmission methods. Information transmission has shifted from the era of writing to the era of reading pictures, and traditional media have shown obvious disadvantages in the protection and dissemination of intangible cultural heritage. Information visualization not only gives people a new experience but also makes people more pleasant and more engaged and allows viewers to gain insight into more information. At the same time, it can provide protection for the inheritance and dissemination of intangible cultural heritage and make the inheritance of intangible cultural heritage more artistic, communicative, and educational [1].

In this big environment, it is still very difficult to efficiently find, understand, and analyze information connections [2]. Visualization can transform obscure and complicated information content into simple and easy-to-read information graphics through visual methods, which greatly improves the efficiency of information acquisition. In the era of global diversification and informatization, it is a very effective and practical way to use digital technology to protect and inherit national intangible cultural heritage [3].

## 2. Literature Review

Conrad et al.'s book series “Virtual Reality Basic Course” proposes that dynamic environment modeling will become a bridge between the real environment and the virtual environment [4]. Integrate decentralized virtual reality systems to build a new virtual system that matches each other in time and space, which is convenient for participants to use and experience. Toktas and O'Neal in the journal *The Application of Virtual Reality Technology in the Protection and Inheritance of Intangible Cultural Heritage* proposed that intangible cultural heritage culture is inherited between families, teachers and apprentices, and ethnic groups, the communication method is very limited, and the use of virtual reality technology is in line with the development of the times and can attract more young people to experience and learn intangible cultural heritage [5]. Yang et al. in the “Research Review of the Application of Virtual Reality Technology in Tourism Abroad” proposed to use virtual reality technology to revive it and reproduce a certain place's heyday society through virtual images [6]. Zi-Jun et al. used 3D scanning and modeling technology to store and apply traditional Chinese medicine knowledge for the first time in “Research and Application of Acupuncture Tongren 3D Visualization” and developed acupuncture Tongren interactive system, which realized TCM visual interactive query of acupoints, meridians, and common diseases [7]. The team led by Lei et al. solved the problems of functional module analysis, model establishment, scene import, and sky box addition of the scenic 3D roaming system and established a 3D interactive roaming system for scenic spots [8]. Yuan et al. used AutoCAD, 3dsmax, Photoshop, and other software to design the virtual hometown scene and finally realized the human-computer interaction functions such as season selection, scene roaming, and information interaction in Unity3D [9]. Aokage et al. pointed out in the analysis of the network influence factor (WIF) that the internal links of websites are often centered on navigation; if a website is large in scale, the number of internal links will increase accordingly, and the importance of the website cannot be judged [10]. Therefore, they adjusted the network impact factor (WIF): if the target “*A*” is at a specified time, after excluding the number of pages of “*A*” itself, the number of web pages linked to a website or a certain area on the Internet, if *Z* is used to represent, that is, *Z* is the number of external links, and the number of web pages of this website or area is expressed as *y*, then the network impact factor of “*A*” is WIF = *z*/*y*.

On the basis of current research, the author proposes a variety of research methods, such as literature reading, actual historical research, case study, and practical research, combined with Xiuyu craftsmanship. Using the method of interdisciplinary research, the author uses computer science, pedagogy, human-computer interaction technology, and simulation technology to conduct cross-disciplinary research and organically combines his research theories for the study of this topic. Using the historical research method, the origin of nonhereditary inheritance is explored in detail, and the longitudinal time comparison of inheritance is carried out. By using the case study method, by comparing the domestic and foreign intangible cultural heritage measures, the method and methods of virtual reality applied to the inheritance and dissemination of intangible cultural heritage are investigated. Using the experimental research method, the theoretical guidance of the paper is used as the support point of practice, and case design is carried out to disprove the validity of the theoretical research content. The author fully integrates theoretical research into specific practice and plays a directional guiding role; the practice process and results are summarized and refined to further improve the theory; this method of combining theory and practice makes virtual reality more systematic and scientific in the research of interaction design platforms.

## 3. Methods

### 3.1. Visual Content

#### 3.1.1. Visual Content and Direction Sorting

Intangible cultural heritage has multiple attributes, including temporal attributes (such as birth year and approval year), spatial attributes (such as birthplace and place of circulation), relationship attributes (including inheritance), hierarchical attributes, people-related attributes, and multidimensional synthesis attributes (such as spatiotemporal multidimensional attributes); it is suitable for visualization by combining time-based visualization methods (such as time series diagrams and calendar diagrams), geographic information-based visualization methods (such as GIS), hierarchical information visualization, and multidimensional visualization methods in the visualization discipline [11]. In order to dig out the feasible visualization direction and content, in-depth interviews were conducted with experts in the field of intangible cultural heritage and visualization, and the following research directions were summarized: (1) Time sequence diagram of the development of intangible cultural heritage: it reflects the evolution of the whole or part of the intangible cultural heritage list at different time stages in chronological order and can clearly see the production sequence and evolution law of intangible cultural heritage. (2) Intangible cultural heritage heat map: describe the intangible cultural heritage items, perform keyword search, get the search popularity according to the search results, and determine the heat value according to color, size, orientation, etc. (3) Intangible cultural heritage relationship diagram: describe the relationship between the intangible cultural heritage items and use the relationship between different nodes to represent the relationship between the intangible cultural heritage items, such as derivative relationship and joint relationship. (4) Intangible cultural heritage and region: the classic mode in the visualization map, which combines intangible cultural heritage attributes with space, describes the overall information of intangible cultural heritage in space and grasps the geographical location of intangible cultural heritage through the map. (5) Nongenetic inheritance relationship diagram: use the relationship between nodes and nodes in the relationship diagram to describe the relationship between the inheritors; the relationship line can be undirected or directional, such as the relationship between master and apprentice, father and son, and brother and sister. (6) Detailed introduction map of key intangible cultural heritage: decompose and reconstruct a single intangible cultural heritage item, interpret key and hot items in detail, and use interesting forms or storylines to express the data readability.

#### 3.1.2. Create a Metadata Database

Refer to the formulation standards of international metadata databases, such as CDWA, a database of artworks and digital image resources, and VRA, a database of art and folk culture, in order to determine the attributes of the intangible cultural heritage metadata database. The intangible cultural heritage database attributes are determined as general attributes and core attributes [12]. The core attributes include the basic information of intangible cultural heritage such as name, type, batch, and application area. The general attributes include more than 30 items such as inheritance method, distribution, subject matter, derivation, and origin; for example, the Softmax classifier is based on the Softmax classifier connection, the deep convolutional neural network can classify and process specific target objects, and based on the classification to fully popularize the logistic regression model, the Softmax regression is obtained [13]. The labeled *m* samples constitute the logistic regression training set. In formula {(*x*^(1)^, *y*^(1)^), ⋯, (*x*^(*m*)^, *y*^(*m*)^)}, *x*^(i)^ ∈ *R*^*n*+1^ is the input feature. *n* + 1 is the *x* dimension of the feature vector, and *x*_0_ = 1 corresponds to the intercept term. Because binary classification is the goal of logistic regression, there is *y*^(*i*)^ ∈ {0, 1}. If the following functions exist,

(1) $$\begin{array}{c} h_{\theta }=\frac{1}{1+\exp\left(-\theta^{T}x\right)}. \end{array}$$

Train the model parameters, which are essentially functions that allow it to minimize the loss:

(2) $$\begin{array}{c} J\left(\theta \right)=-\frac{1}{m}\left[\overset{m}{\underset{i=1}{\sum }}y^{\left(i\right)}\log h_{\theta }\left(x^{\left(i\right)}\right)+\left(1-y^{\left(i\right)}\right)\log\left(1-h_{\theta }\left(x^{\left(i\right)}\right)\right)\right.. \end{array}$$

The number of *y* (category labels) values is different *k*, mainly because it is a multiclassification problem that needs to be dealt with. So, for {(*x*^(1)^, *y*^(1)^), ⋯, (*x*^(*m*)^, *y*^(*m*)^)}, there are (*i*) ∈ {1, 2, ⋯, *k*} class labels, and for a sample input (given) *X*, the probability *p*(*y* = i|*x*) of each classification result can be represented by a *k*-dimensional vector output.

### 3.2. Implementation of Virtual Reality Technology in Xiuyu Craftsmanship

The conventional methods of acquiring images are usually cameras, video cameras, scanners, etc. What these means only acquire is the two-dimensional image of the scanned object, that is, the two-dimensional plane information of the outline of a single side. At present, more and more 3D scanning technologies have replaced the previous scanning methods, made up for the shortcomings of 2D scanning in spatial data, and can accurately reflect the data information of entities in real space [14]. A 3D scanner is a scientific instrument used to detect and analyze the shape (geometric structure) and appearance data (such as color and surface albedo) of an object. It can accurately obtain the three-dimensional coordinates and three-dimensional digital model of the outer surface of the object in space. 3D scanning technology has now developed into the fourth generation of handheld scanning technology [15]. For the collection of the original model of the jade, the complete data of the jade can be obtained by using a handheld laser scanner. It has the characteristics of precision, efficiency, flexibility, and ease of use. The scanner and the computer update the recorded data in real time through the data interface, which provides a basic guarantee for the further processing of jade.

The virtual reality design includes five parts: designing, cutting, carving, polishing, and outputting the scanned jade model. First, analyze the scanned jade from multiple angles, design the model through two-dimensional graphics software, use convenient tools such as copying and mirroring to assist in the drawing of drawings, repeatedly adjust the matching degree between the graphics and the jade, then use the MAYA cutting tool to cut the jade, use various brushes in ZBrush to carve the jade model in detail, and increase the subdivision level to achieve the effect of polishing. Finally, the prepared model is imported into Unity3D, and the human-computer interaction interface for editing operations such as displacement, rotation, and scaling is further set up [16].

In the jade processing process, virtual technology is used to carry out specific operations such as design, simulation, modeling, and interaction, and the product modeling, cost, process, and other aspects are simulated in advance; it not only brings predictability to jade processing but also adds more artistic creativity. The virtual reality design model has absolute advantages; especially for jade processing with excellent raw materials, virtual reality technology is particularly important. It has fundamentally changed the characteristics of the traditional production mode, such as being complex, repetitive, and closed. Taking the interactive 3D model in virtual design as the carrier, the design concept and processing process of the craft master are conveyed in a more intuitive way, so that the designer can repeatedly speculate and analyze the beautiful appearance, reasonable structure, and processing technology. Customers can deeply appreciate the value of Xiuyu craftsmanship through immersive viewing. Engraving students can practice the jade carving craftsmanship through virtual reality. As a result, Xiuyan jade carving can be maximized in the fields of creation, processing, production, sales, and training.

### 3.3. Xiuyu Process Flow Based on Virtual Reality Technology

The specific steps of introducing virtual reality technology in Xiuyu processing are shown in Figure 2.

#### 3.3.1. 3D Scan Data Sampling

The image of jade material is converted into a format that can be read, stored, and edited by the computer through 3D scanning. The data sampling is to reproduce the jade material by means of cloud points, so that the outline features of the jade material are virtualized. The cloud point collection can directly generate the block surface structure, section line, etc., of the jade material, which makes the 3D model construction more accurate and convenient, and quickly switches the entity to the computerized digital management mode.

#### 3.3.2. Product Two-Dimensional Graphic Design

Based on three-dimensional scanning, the computer converts the jade in the virtual space into digital graphics and obtains the drawing object of the two-dimensional graphics, so that the design can be targeted. The two-dimensional editing software adopts another digital expression of the outline image of the design graphics; in the two-dimensional design software, the design image is drawn on the two-dimensional coordinate position of the model through the pressure-sensitive pen of the hand-painted board, so as to maximize the use of the whole piece of jade; the material is used for creation; finally, the two-dimensional visual expression graphic information is presented on the computer [17].

#### 3.3.3. Virtual Cutting and Matching of Raw Materials

To map the 2D design image to the main view in the 3D software, in order to avoid stretching after mapping, it is necessary to unfold the UV lines of the jade model in the 3D software in advance. Cut and extrude the model according to the line draft on the stone and further stretch, rotate, zoom, and other three-dimensional algorithms to control the point, line, and surface of the model in three views, symmetrical objects are mirrored and replicated, and finally, a three-dimensional digital display of the jade model in the design drawings is constructed. When operating, it is necessary to combine both the two-dimensional design drawings and the three-dimensional scanning data and constantly try and modify in the most reasonable interactive way to achieve the final effect [18].

#### 3.3.4. 3D Model Carving

After completing the above steps, the computer has stored the basic model parameters of the jade product, but the model at this time is a rough model designed according to the drawings, and the relief and texture in the jade need to be further refined [19]. In the engraving software ZBrush, the rich engraving brushes are used to simulate the effect of various drill bits in the Xiuyu process for processing jade. After the model is made, the subdivision level is increased to achieve the effect of polishing.

#### 3.3.5. Virtual Reality Display

Import the produced jade model into Unity3D for an all-round virtual immersive display.

### 3.4. Digital Data Collection and Digital Model Establishment

#### 3.4.1. Digital Data Collection

In order to obtain more detailed information on Xiuyu, the author went deep into the local area of Xiuyan, conducted a field investigation on the processing technology, and collected relevant information. The main contents include the following: the processing design patterns of Xiuyu are collected, the traditional Xiuyu processing tools are collected, and the digital model of jade is scanned and collected [20]. After the inspection, the materials such as pictures and patterns are further classified, screened and processed, and turned into digital material files required for virtual reality design. The contents of digital collection are shown in Table 1.

#### 3.4.2. Digital Pattern Processing

The evolution of Xiuyu design has evolved from simple patterns in primitive society to rough patterns in slave society, then to exquisite patterns of flowers, birds, fish, insects, birds, and animals and auspicious patterns in feudal society, all of which embody the unique aesthetics of each period. In the interactive design, the platform will provide users with traditional Chinese jade carving patterns and the shapes of Xiuyu plain furnaces, bottles, tripods, and smokes [21]. The collected pictures are processed into outline graphics by the vector software CorelDRAW, which makes the designer's material calling and reference more concise and intuitive.

In the Unity3D engine, the texture space coordinates of the collision point can be ray-detected by using RaycastHit.textureCoord. When users pick brushes or other tools through the VR handle, they can modify the texture space through the ray collision points in the virtual space. Similar to drawing operations, many intersections and UV coordinates of the model's normal map are generated every second. We can modify the bump on the jade surface by fusing the normal map. The original model after jade scanning itself has a flat normal map, and we constantly operate to superimpose the normal map of the engraving point to appear scratches and patterns [22].

## 4. Experimental Results and Analysis

The judgment matrix of the evaluation indicators of the intangible cultural heritage website and the weight and consistency test of each indicator are as follows; after three rounds of expert survey and scoring, the full frequency of the first-level indicators is information content (C1) 100%, website design (C2) 85.71%, website function (C3) 64.29%, website influence (C4) 42.86%, and website security (C5) 21.43%. Based on this, the judgment matrix is constructed and the relative weight is calculated, as shown in Table 2.

According to a big data survey of intangible cultural heritage culture, most users prefer to understand intangible cultural heritage culture through “experience” and feel that personal experience is more intuitive and interesting, as shown in Figure 3. This provides a broad market prospect for virtual intangible cultural heritage experience [23].

The dissemination of intangible cultural heritage information through virtual reality technology through questionnaires enables more people to experience intangible cultural heritage culture; the questionnaire survey shows that more than 60% of more than 1000 people experience intangible cultural heritage culture.

At the same time, a total of 30 users were selected to test the visualization platform; the target audience includes three types of groups: heritage artists, factory apprentices, and college students; the research includes four factors, namely, the interactive performance of the visualization platform, system speed, module experience accuracy, and professionalism technical acquaintance, as shown in Table 3. The test results show that 90% of users are willing to combine jade carving technology with 3D scanning virtual reality technology, and only 15% of the test users have some understanding of virtual technology and 3D scanning technology; it shows that there are few practical cases of 3D scanning virtual technology combined with manual skills, which also increases the difficulty of promoting the visualization platform; in the later stage, it is necessary to further improve the operation performance of the system, reduce the technical difficulty of visualization, and increase the matching degree of technology [24, 25].

## 5. Conclusion

In general, 3D scanning and virtual reality technology have spawned a new concept of subversive visual communication, challenged the traditional static visual communication form, and attracted people's attention and recognition with a more flexible and dynamic form of expression. The research on the visualized Xiuyu platform realizes the function of combining technology and inheritance, breaks the single inheritance mode of traditional skills, and makes the dissemination of traditional skills more efficient. Display and disseminate intangible cultural heritage through digital media and digital platforms and further realize the cultural inheritance of intangible cultural heritage in the digital space. With the rapid development of science and technology, virtual reality technology will definitely become an important way for the inheritance and dissemination of my country's intangible cultural heritage. Due to its digital and virtual nature, it has broken through many limitations in the way of protection and solved the singleness and limitations of traditional intangible cultural heritage protection methods. The intangible cultural heritage graphic database, intangible cultural heritage model database, intangible cultural heritage digital aided design, intangible cultural heritage virtual technology innovation process, etc., will definitely make more contributions to the inheritance and dissemination of intangible cultural heritage in my country.

## Figures and Tables

**Figure 1:** Age distribution of the fifth batch of national nongenetic inheritors.

**Figure 2:** Implementation step diagram.

**Figure 3:** Proportion of participation in intangible cultural heritage.

**Table 1:** Digital collection content.

Collection object	Collect content
Design patterns	Pattern, animal pattern, plant pattern, figure pattern, plain pattern
Machining tools	Jade carving flat knitting machine, jade carving electronic pen, saw blade, grinding head, grinding needle, drill bit
Jade scan	Hemo jade, lao jade, new mountain jade, hua jade, jia cui

**Table 2:** Judgment matrix and weight of first-level indicators in the evaluation system of intangible cultural heritage websites.

	C1	C2	C3	C4	C5	*W*_*i*_ (权重)
C1	1.000	1.369	2.191	3.509	5.618	0.377
C2	0.731	1.000	1.601	2.563	4.105	0.276
C3	0.456	0.625	1.000	1.601	2.564	0.172
C4	0.285	0.390	0.625	1.000	1.601	0.108
C5	0.178	0.244	0.390	0.625	1.000	0.067
Consistency ratio: 0.000	Largest characteristic root: 5.000					

**Table 3:** Experience evaluation of the engraving part of the platform.

Test number	Test items	The proportion
1	Most concerned about the platform engraving part	95%
2	Satisfaction with the engraving part	72%
3	Degree of expectation after modification	85%

## Data Availability

The data used to support the findings of this study are available from the corresponding author upon request.
